The article "Effect of Ultrasonic Osteotome on Therapeutic Efficacy and Safety of Spinal Surgery: A System Review and Meta-Analysis" was published in 2022. Journal: Comput Math Methods Med.

# Effect of Ultrasonic Osteotome on Therapeutic Efficacy and Safety of Spinal Surgery: A System Review and Meta-Analysis

**DOI:** 10.1155/2022/9548142

**Published:** 2022-08-29

**Authors:** Leilei Wu, Sheng Wang

**Affiliations:** Spine Surgery, Affiliated Hospital of Weifang Medical University, 261031, China

## Abstract

**Background:**

A meta-analysis was performed to evaluate the effectiveness and safety of ultrasonic osteotomes in spine surgery to standard spinal surgery procedures.

**Methods:**

Using the search keywords “bone curette”, “cutter”, “scalpel”, “bone shaver”, “aspirator”, “osteotome”, “ultrasonic”, “piezosurgery”, and “dent  ^∗^” in the databases of PubMed (1966-2021.12), Cochrane Library, Embase (1986-2018.12), Web of Science (1978-2021.12), and China Academic Journals Full-Text Database (CNKI, 1979-2021.12). Two researchers reviewed the literature, extracted and extensively assessed the data, and included information on the study quality. RevMan v5.3.5.0 was used for the meta-analysis.

**Results:**

A total of 10 trials with a total of 911 patients were included. The meta-analysis findings revealed that, when compared to traditional methods, ultrasonic osteotomes could save operation time (OR = −18.83, 95 percent CI (-22.76, -14.99), *P* = 0.03) and reduce intraoperative bleeding (OR = −66.73, 95 percent CI (-75.70, -57.76), *P* = 0.04) and postoperative complications (OR = 0.38, 95 percent CI (0.21, 0.69), *P* = 0.001). There was, however, no significant difference in the hospital stay (OR = −1.34, 95 percent CI (-1.90, -0.77), *P* = 0.23) and symptom improvement rate (OR = 1.03, 95 percent CI (0.73, 1.45), *P* = 0.86).

**Conclusion:**

There is evidence that using an ultrasonic osteotome in spine surgery is safe and effective and may minimize intraoperative bleeding and save time. However, there is no significant difference in symptom improvement rate, hospital stay length, or postoperative complications compared to standard surgical equipment. Therefore, more high-quality investigations are needed to corroborate the initial results.

## 1. Introduction

As the human body's second lifeline, the spine is responsible for the central axis bone and nerve conduction of the human trunk and surrounding intricate nerves and blood vessels [1]. Its clinical operation is highly complex and risky, with high demands for preoperative, midoperative, and postoperative image confirmation, surgical equipment, operator experience, and operation technology. Spinal surgery technology has advanced fast due to the advancement of surgical equipment [2]. Although high-speed drills (HSDs), osteotomes, laminectomy forceps, nucleus pulposus forceps, and other traditional surgical instruments in spinal surgery are widely used in intraoperative decompression and osteotomy [3], studies have shown that they can cause intraoperative nerve, blood vessel, spinal cord, dura mater, and other injuries. On the other hand, traditional spinal surgery relies on physicians' clinical knowledge and intraoperative scanning pictures. It thus has several drawbacks, such as substantial trauma and long postoperative recovery [4].

The article "Effect of Ultrasonic Osteotome on Therapeutic Efficacy and Safety of Spinal Surgery: A System Review and Meta-Analysis" was published in 2022. Journal: Comput Math Methods Med.

Piezosurgery is a bone surgery equipment that works on the basis of high-intensity focused ultrasound (cavitation effect, thermal effect, and mechanical effect) [5]. The transducer in the knife converts electrical energy into mechanical energy by using high-intensity focused ultrasound technology [6]. After a high-frequency ultrasonic vibration, the water in the contacting tissue cells evaporates and the protein hydrogen bond is destroyed, fully damaging the bone tissue to be cut during the surgery [7]. The ultrasonic cutter head operates at a temperature of less than 38°C and a propagation distance of less than 200 microns [8]. Because high-intensity focused ultrasound can only destroy bone tissue of a certain hardness, it does not harm blood vessels or nerve tissue while also stopping bleeding at the surgical wound, reducing the impairment of minimally invasive surgery, and significantly improving accuracy, reliability, and safety. It is currently widely used in oral and maxillofacial surgery. Hidaka employed UBC in a cervical double-door laminoplasty for the first time in 1998, indicating that it may reduce the risk of intraoperative nerve and dural injury. Since then, UBC has piqued the interest of a growing number of spine surgeons [9].

In recent years, there has been an increase in the number of reports on the use of UBC in spine surgery. However, because of the small number of cases and lack of data, there is still no consensus on UBC's effectiveness and safety [10]. As a consequence, this study collected relevant literature comparing the effectiveness and safety of UBC and traditional tools in spinal surgery in the United States and overseas for meta-analysis in order to provide evidence-based medical data supporting the use of UBC in spinal surgery.

## 2. Materials and Methods

### 2.1. Search Strategy

Search the databases of PubMed (1966-2021.12), Cochrane Library, Embase (1986-2018.12), Web of Science (1978-2021.12), China Academic Journals Full-Text Database (CNKI, 1979-2021.12), Wanfang Database (1998-2021.12), and Google Scholar (1989-2021.12), among other databases. “Bone curette”, “cutter”, “scalpel”, “bone shaver”, “aspirator”, “osteotome”, “ultrasonic”, “piezosurgery”, and “dent  ^∗^” are the English search phrases. All databases have a retrieval period that runs from the moment the database was established until December 30, 2021. In addition, additional references were manually obtained in order to incorporate all of the literature.

The article "Effect of Ultrasonic Osteotome on Therapeutic Efficacy and Safety of Spinal Surgery: A System Review and Meta-Analysis" was published in 2022. Journal: Comput Math Methods Med.

### 2.2. Inclusion and Exclusion Criteria

The inclusion criteria are as follows. (1) The research was intended as a controlled clinical trial of UBC in spinal surgery, involving a randomized controlled study, a cohort study, and a case-control study. (2) The participants included patients having spinal surgery for conditions such as cervical spondylosis, ossification of the thoracic ligamentum flavum, lumbar disc herniation, and lumbar spinal stenosis; spinal trauma; spinal infection; spinal tumor; and spinal deformity; and so on. (3) The experimental group employed UBC to decompress and osteotomize the bone tissue and calcified tissue, whereas the control group used standard surgical tools such as HSD, bone biting forceps, and bone knife. (4) Outcome variables included operation duration, intraoperative bleeding, hospital stay, postoperative neurological improvement, and safety indicators, as well as postoperative sequelae. The criteria for exclusion are as follows: (1) research with less than five examples; (2) overviews, conference papers, and expert opinions; (3) non-English literature; and (4) documents unable to extract data and so on.

### 2.3. Study Selection and Data Extraction

According to the PRISMA flow chart, the first and second authors will undertake screening, literature quality review, and data extraction based on the inclusion and exclusion criteria before conducting the cross inspection. In the event of a dispute, they will be sent to third-party arbitration, with the appropriate author appointed as the third-party arbiter. During the screening process, the authors first use the literature management software to import the title, eliminate the repetition, and then browse the label to exclude the literature not related to this study. If the information contained in the title is insufficient to exclude, the method of reading the abstract and full text shall be used to determine whether it can be included. If necessary, the authors attempt to contact the original research author through email or phone to collect data information that has not yet been identified but is critical for this investigation. A predesigned data extraction form is used for recording. The specific components are as follows: (1) the title of the article included in the study, the original author, the publication date, and the magazine in which it was published; (2) subject baseline characteristics and intervention measures for the experimental and control groups: sample size, gender, age, disease course, classification, intervention technique, length of treatment, withdrawal, follow-up, and so on; (3) relevant aspects of bias risk assessment: adherence to the randomization principle, blindness, dispersion and concealment, and so on; and (4) measurements of outcome, including main and secondary: incision time, bleeding volume, postoperative JOA, complications, and so forth.

The article "Effect of Ultrasonic Osteotome on Therapeutic Efficacy and Safety of Spinal Surgery: A System Review and Meta-Analysis" was published in 2022. Journal: Comput Math Methods Med.

### 2.4. Bias Risk Assessment

The risk of bias was assessed and cross-checked by the first and second authors using the inclusion and exclusion criteria. Any issue must be resolved via arbitration with a third party. The risk of bias in RCT studies was assessed using the Cochrane Library's suggested technique, while the risk of bias in cohort studies was assessed using the NOS grading scale.

### 2.5. Statistical Analysis

The data in the study were meta-analyzed using RevMan software v5.3.5.0. If the information is of the counting type, the combined statistics are relative risk (RR) or odds ratio (OR); if it is of the continuous variable type, the weighted mean difference (WMD) is used for meta-analysis, and the 95 percent confidence interval (CI) is presented. In addition, use 2. Perform a heterogeneity test. If *P* > 0.10 and *I*^2^ > 50, analyze heterogeneity using the fixed effect model, followed by a source of heterogeneity analysis and subgroup analysis depending on the causes for heterogeneity. If the heterogeneity cannot be decreased or the *I*^2^ is more than 50, the random effect model is employed to analyze the data. Furthermore, if the heterogeneity is too great and lacks analytical significance, a descriptive analysis will be performed. Set the significance criterion for meta-analysis to = 0.05. When the number of the included pieces of literature surpassed 10, an inverted funnel diagram was used to analyze the publication bias of the included research.

## 3. Results

### 3.1. Research Characteristics

In all, 920 pieces of relevant literature were gathered. Following the screening, ten studies with a total of 911 participants were chosen, including five randomized controlled trials and five cohort studies. The document screening method is shown in Figure 1.  Table 1 summarizes the key elements of the included investigation.

### 3.2. Data Quality Assessment

The bias risk assessment found that the one randomized controlled trial had significant levels of selection bias, implementation bias, and measurement bias, as well as poor overall quality. One of the five cohort studies assessed received a NOS score of 6, two received a score of 7, and two received a score of 8. The overall quality of the cohort research was outstanding (Figure 2).

The article "Effect of Ultrasonic Osteotome on Therapeutic Efficacy and Safety of Spinal Surgery: A System Review and Meta-Analysis" was published in 2022. Journal: Comput Math Methods Med.

### 3.3. Operation Time of Patients

The operation time was recorded in ten trials. The heterogeneity test findings were *P* < 0.00001 and *I*^2^ = 51%. The random effect model was used for meta-analysis. As shown in Figure 3, the findings revealed that the mean operating time (min) of the UBC group was shorter than that of the traditional surgical method group, and the difference was statistically significant (OR = −18.83, 95 percent CI (-22.76, -14.99), *P* = 0.03).

### 3.4. Intraoperative Bleeding in Patients

Five research reported on the quantity of intraoperative bleeding. The heterogeneity test findings were *P* < 0.00001 and *I*^2^ = 59%. The random effect model was used for meta-analysis. As demonstrated in Figure 4, the quantity of intraoperative bleeding in the UBC group was smaller than that in the traditional surgical method group, and the difference was statistically significant (OR = −66.73, 95 percent CI (-75.70, -57.76), *P* = 0.04).

### 3.5. Hospitalization Time of Patients

The duration of hospital stay was reported in six trials. The heterogeneity test findings were *P* < 0.000 01 and *I*^2^ = 27%. The random effect model was used for meta-analysis. As indicated in Figure 5, there was no significant difference in the duration of hospital stay between the UBC group and the traditional surgical method group (OR = −1.34, 95 percent CI (-1.90, -0.77), *P* = 0.23).

### 3.6. Postoperative Symptom Improvement Rate

Eight studies found that less of the postoperative symptoms improved. The heterogeneity test findings were *P* = 1.00 and *I*^2^ = 0%. For meta-analysis, the fixed effect model was utilized. As demonstrated in Figure 6, there was no significant difference in the rate of improvement of postoperative symptoms between the UBC group and the traditional instrument group (OR = 1.03, 95 percent CI (0.73, 1.45), *P* = 0.86).

### 3.7. Postoperative Complications

A total of ten studies compared patients' postoperative problems. The heterogeneity test findings were *P* = 0.97 and *I*^2^ = 0%. For meta-analysis, the fixed effect model was utilized. As demonstrated in Figure 7, there was a significant difference in the incidence of postoperative problems between the UBC group and the conventional instrument group (OR = 0.38, 95 percent CI (0.21, 0.69), *P* = 0.001).

### 3.8. Publication Bias

A funnel chart was used to explore publication bias. In comparing the postoperative complications of patients in the UBC group and the traditional instrument group, there was no obvious asymmetry in the funnel chart, suggesting no obvious publication bias, as shown in Figure 8.

The article "Effect of Ultrasonic Osteotome on Therapeutic Efficacy and Safety of Spinal Surgery: A System Review and Meta-Analysis" was published in 2022. Journal: Comput Math Methods Med.

## 4. Discussion

Spinal disorders have risen steadily in recent years [10]. However, due to severe fatigue, the cervical and lumbar segments often produce hypertrophy and ossification of the posterior longitudinal ligament and ligamentum flavum [11]. Conventional spinal surgery, such as laminoplasty, uses the “bowstring effect” formed by the spine's physiological lordosis and kyphosis to contact the pressor of the spinal cord or open the space behind the spinal cord to keep the spinal cord from compression and achieve the effect of decompression [12]. Traditional resection primarily employs LP and HSD [13]. Although they have excellent benefits when used correctly, the average vertebral incision duration and the frequency of associated problems are considerable [14]. They have a more precise cutting ability, and the heat energy created by friction with bone tissue during osteotomy may cause hemostasis. Still, the accumulated heat is difficult to grasp, and a too-high temperature can burn the osteotomy's perimeter [15]. Hence, drip cooling is often employed in clinical settings, although studies demonstrate that it cannot diminish the heat effect created by friction. Finally, a response force is made on the handle during the high-speed rotation of the drill bit. Slippage and catastrophic accidents are easily caused by improper operation [16].

The introduction of UBS as a novel osteotomy dynamic system gives spine surgeons a new option. It may selectively cut tissue based on density and elasticity using the rupture and cavitation effects to prevent unintended harm [17]. According to Sanborn et al., the bleeding volume of UBS is smaller than that of LP. UBS is also more secure and dependable than HSD. It has two modes: “regular” and “cold cutting.” The former is suitable for separating soft tissue and bone cortex, has a greater temperature, and may halt bleeding; the latter is very safe when used near the dura mater and spinal cord [18].

Furthermore, rotating the cutting section of UBS on a frequent basis, lengthening the residence time at the same place by 10s, and improving local perfusion may reduce the temperature of the cutting interface, preventing thermal injury [19]. The ability of UBC to minimize operating time has long been a subject of contention among spine surgeons. Some specialists believe that when removing a significant amount of bone or calcification, UBC is less efficient than standard instruments (such as HSD and lamina rongeur) and that the learning curve for UBC is longer. As a consequence, UBC requires more time to operate than ordinary instruments. Most studies now believe that UBC may significantly reduce intraoperative bleeding when compared to typical surgical equipment [20].

The article "Effect of Ultrasonic Osteotome on Therapeutic Efficacy and Safety of Spinal Surgery: A System Review and Meta-Analysis" was published in 2022. Journal: Comput Math Methods Med.

However, according to a research published in 2014 by Byron, which evaluated the efficacy of UBC and HSD in decompression surgery in individuals with achondroplasia, there is no significant difference in hospital stay between the UBC and HSD groups [21]. Our research is partly in line with the results of this experiment, but there are also differences. According to the findings of this meta-analysis, there was no significant difference in hospital stay between UBC and conventional equipment [22]. We feel the following causes are possible. (1) The illness diagnosis of the included individuals varies and is diverse. (2) The baseline levels of patients included in relevant research vary. Most studies employ UBC in patients who have a protracted decompression or osteotomy stage, severe spinal cord compression, and a significant risk of vascular and nerve damage. (3) Each research has a modest sample size [23]. In terms of symptom improvement, two studies in this meta-analysis found no difference between the UBC group and the conventional device group. Eight research studies found that patients' symptoms in the UBC group improved considerably. We feel the following causes are possible: (1) the assessment criteria for symptom improvement in various research varied, (2) the follow-up duration was brief, and (3) the sample size is insufficient.

Bagga et al. believe that the problems in the UBC group are lower than those in the conventional instrument group based on noncontrolled trials [24]. They think this is due to UBC's selective bone cutting and slight injury to peripheral blood vessels and nerve tissue. According to this meta-analysis [25], the incidence of UBC-related complications during spinal surgery was 5.88 percent (12/204), with dural rupture being the most prevalent, accounting for 4.90 percent (10/204). According to the numerous studies, the primary causes of a dural tear include dural ossification or extreme compression, inability to absorb vibration, UBC absorption, involvement, high force, or thermal damage induced by long-term residence [26]. According to the findings of this meta-analysis, there was a statistically significant difference in the incidence of postoperative complications between UBC and conventional tools [27]. We feel the following causes are possible: (1) various physicians' competency in UBC, (2) differences in UBC of different brands, and (3) integrity and validity of medical records.

## 5. Limitations

The study's shortcomings are as follows. (1) There are few high-quality clinical control study papers among the 10 included studies, which include publication bias and selection bias. (2) The research solely includes 911 occurrences. However, there is a substantial gap between patients and the massive sample size and multicenter data required for statistical analysis of evidence-based treatment. (3) There are differences in the ages and diagnoses of the people included in the study, as well as variability throughout the study. (4) It is difficult to identify the details of each research execution, such as whether other traditional instruments (such as curettes) are used in combination with UBC, how skilled doctors are, and how authentic and comprehensive medical records are. As a consequence, it is hard to thoroughly examine UBC's effectiveness and safety and the meta-result analysis should be considered seriously.

The article "Effect of Ultrasonic Osteotome on Therapeutic Efficacy and Safety of Spinal Surgery: A System Review and Meta-Analysis" was published in 2022. Journal: Comput Math Methods Med.

## 6. Conclusion

In conclusion, based on the existing clinical data, using an ultrasonic osteotome in spine surgery is safe and prosperous, reducing intraoperative bleeding and shortening the operation time. However, it offers no clear benefits over standard equipment in easing patients' symptoms, shortening hospital stays, and lowering surgical complications. However, because of the low quantity and quality of the included research, the results mentioned above must be supported by more high-quality investigations.

## Figures and Tables

**Figure 1:** Document screening process.

**Figure 2:** Document quality evaluation.

**Figure 3:** Operation time comparison.

**Figure 4:** Intraoperative bleeding comparison.

**Figure 5:** Hospitalization time comparison.

**Figure 6:** Postoperative symptom improvement comparison.

**Figure 7:** Postoperative complication comparison.

**Figure 8:** Publication bias comparison.

**Table 1:** Literature features included in the study.

Author (year)	Participants	Outcomes
Williams BJ, 2011	78	Provided general benchmarks of durotomy rates and served as a basis for ongoing efforts to improve safety of care.
Street JT, 2012	942	Identified a very high rate of previously unrecognized postoperative complications, which adversely affect LOS. Without strict adherence to a prospective data collection system, the true complexity of this surgery may be greatly underestimated.
Onen MR, 2015	46	For patients with CSM, laminectomy using the UBS provides a safe, rapid, and effective decompression with lesser blood loss. The low rate of complications lessens the postoperative morbidity rates and shortens hospital stay.
Bydon M, 2014	30	Decreased incidence in intraoperative durotomy and overall perioperative complication rates in the BoneScalpel cohort, although this did not reach the level of statistical significance. Nonetheless, the data demonstrate that the BoneScalpel is a safe and efficacious alternative to the high-speed drill in these challenging patients.
Bartley CE, 2014	20	The use of an ultrasonic bone scalpel to perform the bone cuts associated with facetectomies and apical Ponte-type posterior releases resulted in significantly less bleeding compared with cuts made with standard osteotomes and rongeurs, limiting overall blood loss by 30% to 40%.
Bydon M, 2013	337	The safety and efficacy of ultrasonic bone curettes in spine surgery has not been well established. This study shows that the ultrasonic bone curette has a similar safety profile compared with the high-speed drill, although both are capable of causing iatrogenic dural tears during spine surgery.
Matsuoka H, 2012	33	The ultrasonic bone curette is a useful instrument for recapping hemilaminoplasty in various spinal surgeries. This method allows anatomical reconstruction of the excised bone to preserve the posterior surrounding tissues.
Hazer DB, 2016	307	We recommend this device as an assistant tool in various spine surgeries and as a primary tool in foraminotomies. It is a safe device in spine surgery with very low complication rate.
Hu X, 2013	128	Overall, the ultrasonic scalpel was safe and performed as desired when used as a bone cutting device to facilitate osteotomies in a variety of spine surgeries. However, caution should be taken to avoid potential thermal injury and dural tear.
Ito K, 2009	12	The scalpel-type ultrasonic bone curette is useful for cutting bone and effective for the reconstruction of the laminae. Laminotomy with an ultrasonic bone curette is safe and minimally invasive.

The article "Effect of Ultrasonic Osteotome on Therapeutic Efficacy and Safety of Spinal Surgery: A System Review and Meta-Analysis" was published in 2022. Journal: Comput Math Methods Med.

## Data Availability

The datasets used during the current study are available from the corresponding author on request.
